# The Impact of Improved Oral Care Methods on the Oral Health of Patients Undergoing Transoral Mechanical Ventilation

**DOI:** 10.1155/2022/7596654

**Published:** 2022-09-16

**Authors:** Yijun Shen, Ling Dai, Yanwen Zhu, Yishu Lang

**Affiliations:** ^1^Department of Stomatology, Community Health Service Center, Huangyan District, Zhejiang, China; ^2^Wuhan No. 1 Hospital, ICU, China; ^3^Community Health Service Center, China

## Abstract

**Objective:**

To explore the effects of improved oral care on the number of oropharyngeal bacteria and the incidence of ventilator-associated pneumonia in patients undergoing mechanical ventilation through oral endotracheal intubation by improving conventional oral care methods and operating procedures and to evaluate the quality of improved oral care and effect.

**Methods:**

A total of 100 cases of mechanically ventilated patients with oral endotracheal intubation who met the inclusion criteria were randomly divided into the observation group and control group with 50 cases each. The control group took routine oral care, that is, scrubbing 3 times per day, and the oral care solution was selected as physiological brine. The observation group improved the conventional oral care method, namely, oral scrubbing before intubation, brushing and washing after intubation, 3 times per day, and 0.1% povidone-iodine in oral care solution. Analysis and comparison of the oral bacterial flora, oral cleanliness, and incidence of ventilator-associated pneumonia, mechanical ventilation time, ICU hospitalization time, and mortality rate of the two groups of patients were analyzed and compared. The relevant data were collected and processed for statistical processing.

**Results:**

The oral bacterial flora of the two groups of patients before oral care after mechanical ventilation after oral tracheal intubation was compared, and there was no significant statistical difference (*P* > 0.05). After nursing, the oral bacterial flora of the observation group at 8 h, 16 h, and 24 h after intubation was significantly lower than that of the control group. Statistics showed that the difference was statistically significant (*P* < 0.05). After nursing, the number of patients with oral cleanliness in the observation group was significantly higher than that of the control group, while the incidence of ventilator-associated pneumonia in the observation group was 8% significantly lower than that of the control group 14%. Statistics show that this difference is statistically significant (*P* < 0.05). After nursing, the observation group's oral cleanliness score, mechanical ventilation time, ICU hospitalization time, and GCS score were better than those of the control group. Statistics showed that the difference was statistically significant (*P* < 0.05). The mortality of the observation group was significantly lower than that of the control group, which was not statistically significant (*P* > 0.05).

**Conclusion:**

Oral care can effectively reduce the number of oropharyngeal bacteria in patients who are mechanically ventilated through orotracheal intubation and significantly reduce the incidence of ventilator-associated pneumonia.

## 1. Introduction

Mechanical ventilation through airway intubation is an important measure to save the life of patients with respiratory failure. Patients with mechanical ventilation will have a series of oral complications after catheterization, including changes in oral pH value, changes in the composition and function of saliva, disorders of cough and swallowing, changes and displacement of oropharyngeal colonization bacteria, and increase of dental plaque [1]. Mechanically ventilated patients cannot eat through the oral cavity, which leads to a decline in the self-purification function of the oral cavity. The secretions accumulate and sink around the balloon of the tracheal tube. Bacteria can easily enter the bronchopulmonary tissue and cause lung infection [1]. Ventilator-associated pneumonia is an important type of hospital-acquired pneumonia, and it is a common and dangerous complication in assisted ventilation patients [2]. Imperfect immune development can lead to more likely lung infections during assisted ventilation; in addition to the small size of the patient's mouth, oral care is more difficult, and nurses tend to neglect the care of the oral cavity [3].

At present, for patients with endotracheal intubation, most nursing staffs carry out oral care according to experience and habit, and the level of oral care of nursing staff and mechanical ventilation patients' oral care effect is uneven. The comprehensive evaluation system of oral care is the premise and basis for the implementation of effective oral care, but because there is no system, the evaluation of patients with tracheal intubation is feasible in nursing staff according to the patients with local oral intubation time, condition, and situation, especially the oral microbial species choosing appropriate oral care methods and pertinence of oral care solution and local drug use. The implementation of individualized and diversified oral care greatly affects the quality of oral care for intubation patients, as well as the effectiveness of oral care, which is a safe, effective, economic, and convenient measure to prevent the occurrence of ventilator-associated pneumonia and improve the quality of oral care for intubation patients [4]. Therefore, this study explores the impact of improved oral care methods on the oral health of patients undergoing oral mechanical ventilation and provides a reference basis for the clinical care of mechanical ventilation through oral endotracheal intubation.

## 2. Information and Methods

### 2.1. Research Object

The medical records of 100 patients who were treated and nursed in our hospital from March 2018 to March 2021 who received mechanical ventilation through oral endotracheal intubation were selected as the research objects and were randomly divided into the observation group and control group with 50 cases each. In the observation group, there were 28 males and 22 females, aged 21-83 years old, with an average of 61.98 ± 11.2 years old. Disease composition is as follows: 22 cases of the respiratory system, 18 cases of the circulatory system, 4 cases of the nervous system, and 6 cases of the urinary system; dental condition of patients is as follows: 24 cases had teeth and 26 cases had no teeth. In the control group, there were 24 males and 26 females, aged 23-81 years old, with an average of 58.62 ± 7.2 years old. Disease composition is as follows: 21 cases of the respiratory system, 19 cases of the circulatory system, 4 cases of the nervous system, and 6 cases of the urinary system; dental condition of patients is as follows: 23 cases had teeth and 27 cases had no teeth. The baseline data such as age and gender of the two groups of patients were not statistically significant (*P* > 0.05). All patients and their families signed informed consent.

### 2.2. Inclusion and Exclusion Criteria

Inclusion criteria were as follows: (1) patients with ventilator-associated pneumonia meet the diagnostic criteria of the “Guidelines for the Diagnosis, Prevention and Treatment of Ventilator-Associated Pneumonia (2013)” [5]; that is, use a ventilator for >48 hours or weaning and extubation within 48 hours, new or progressively enlarged lung infiltrative shadows appeared on chest X-ray or chest CT, and one of the following conditions was met at the same time: lung consolidation signs and/or pulmonary wet rales, the total number of peripheral blood white blood cells increased (WBC > 10.0 × 10 L), fever, purulent secretions of the respiratory tract, and new pathogenic bacteria were cultivated from the secretions. The patient has a clear consciousness and can speak normally; (2) ICU patients who require mechanical ventilation via oral tracheal intubation, aged ≥18 years, and mechanical ventilation time ≥ 14 days; (3) all collected clinical data are complete; (4) the clinical information of the patients in this study must be complete. Exclusion criteria were as follows: (1) patients with severe bleeding, coagulation dysfunction, and iodine allergy; (2) patients with heartbeat, respiratory arrest, or other emergency tracheal intubation, oral surgery, and severe respiratory burns; and (3) patients with oral diseases, lung infections, and contraindications for semirecumbent position.

### 2.3. Method

According to ICU routine care and tracheal tube care, in posture nursing, the patient takes a 3 ~ 45° semirecumbent position, and closed sputum suction nursing is as follows: nursing care of airway humidification and care of ventilator pipes, that is, cotton ball wipes 3 times, 8 hours apart, and timed from the tracheal intubation, and the oral care solution is normal saline.

#### 2.3.1. Routine Oral Care

(1) According to the routine oral care scrub method, here is the order of scrubbing: the outer surface of the upper dentition, the inner surface, the occlusal surface, the outer surface of the lower dentition, the inner surface, the occlusal surface, and then the cheeks are scrubbed in an arc shape. (2) Take the regular oral care scrubbing method, namely, cotton ball scrubbing method 3 times, and 8 h interval timing when intubation from trachea. Oral care solution uses physiological saline.

#### 2.3.2. Improved Oral Care Model

(1) Oral scrub before intubation is as follows: use 0.1% povidone-iodine gauze block to scrub the oral cavity once (completed within 2 minutes). The order of scrubbing is the outer surface⟶the inner surface⟶the occlusal surface⟶the cheek⟶the tongue surface. (2) Put the children's soft bristled toothbrush into 0.1% povidone-iodine solution and soak for 15 s to soften the bristles. Brush the inside and outside of the teeth vertically and the teeth on the occlusal surface horizontally. The order of brushing is the outer surface⟶the inner surface⟶the occlusal surface⟶the cheek⟶the tongue surface. (3) Raise the head of the bed 20~ 30°C, check the balloon pressure in the tracheal tube (balloon pressure 25~ 35 cmH2O), record the depth of the intubation to the incisor, and fully absorb the secretions in the respiratory tract and oral cavity. Here are the following examples operated by two nurses: one nurse fixes the patient's head and intubation with one hand, moves the tracheal tube to one side of the mouth, and draws 0.1% povidone iodine with a syringe in the other hand and treats the patient's teeth, cheeks, and cheeks from different directions. The tongue, throat, and palate were rinsed, and another nurse sucked out the rinse with a suction tube from the corner of the patient's other mouth. Repeatedly, until the mouth was rinsed clean

### 2.4. Observation Indicators

① Oral bacterial flora was as follows: the throat swab specimens are collected by the fixed personnel according to the conventional specimen collection method, respectively, 8 h, 16 h, and 24 h after intubation, and 30 min before and after oral care. After intubation, the secretions were collected around both sides of the palatal arch, pharynx, and tonsils (the specimens were sent for examination within 30 minutes). ② Oral cleanliness score was as follows: evaluate the status of oral hygiene. The oral cleanliness scoring method was as follows: “Basic Nursing” Oral Nursing Evaluation Form (People's Medical Publishing House, Fourth Edition). There are 12 items in total, each of which means 1 means “good,” 2 means “fair,” and 3 means “bad,” and the total score is 12-36 points. The higher the score, the more oral hygiene is needed. Care. VAP incidence rate (%): number of selected cases with VAP/total number of selected cases, mechanical ventilation time (d): from the mechanical ventilation of the tracheal intubation to the end of the mechanical ventilation, ICU hospital stay (d): the number of days from admission to ICU, and mortality rate (%): death toll of selected cases/total number of selected cases. Cronbach's *α* values measured on the above scales before use were all greater than 0.914. The patient fills in independently without being affected by any internal or external factors, and the test will be completed within 30 minutes.

### 2.5. Statistical Methods

Use EpiData to enter all the data and then use SPSS 25.0 to statistically process the data. The data needs to be entered into the computer database by a second person to ensure the completeness and accuracy of the data. Use *t*-test or repeated measures analysis of variance to express the measurement data as mean ± standard deviation ($\bar{x}\pm S$) and use the *χ*^2^ test to express the count data as percentage (%), with statistical significance *P* < 0.05.

## 3. Results

### 3.1. Comparison of Oral Bacterial Flora

The oral cavity is scrubbed within 30 minutes before intubation to strengthen oral cleaning before intubation Figure 1. The oral bacterial flora of the two groups of patients before oral care after mechanical ventilation and after oral tracheal intubation was compared, and there was no significant statistical difference (*P* > 0.05). After nursing, the oral bacterial flora of the observation group at 8 h, 16 h, and 24 h after intubation was significantly lower than that of the control group. Statistics showed that the difference was statistically significant (*P* < 0.05), see Table 1.

### 3.2. Comparison of Oral Cleanliness and Incidence of Ventilator-Associated Pneumonia

Aspiration is a common complication of patients during the treatment of mechanical ventilation through oral endotracheal intubation, if the bacteria in the oropharynx reach the lungs through aspiration. After nursing, the number of patients with oral cleanliness in the observation group was significantly higher than that of the control group, while the incidence of ventilator-associated pneumonia in the observation group was 8% significantly lower than that of the control group 14%. Statistics showed that this difference was statistically significant (*P* < 0.05), see Table 2.

### 3.3. Comparison of Mechanical Ventilation Time, ICU Hospitalization Time, and Mortality

This study is aimed at improving the inefficiency and limitations of oral care for patients with clinical oral endotracheal intubation and strengthened early oral cleaning before intubation and oral care after intubation. After nursing, the observation group's oral cleanliness score, mechanical ventilation time, ICU hospital stay, and GCS score were better than those of the control group. Statistics showed that the difference was statistically significant (*P* < 0.05). The mortality of the observation group was significantly lower than that of the control group, which was not statistically significant (*P* > 0.05), see Table 3.

## 4. Discussion

Due to intubation and mechanical ventilation, the dynamic balance of oral flora in mechanically ventilated patients is broken, and the oral flora is reproduced pathologically, which is related to the continuous open state of the oral cavity and airway of mechanically ventilated patients, increased saliva secretion, and the continuous reproduction and accumulation of oral bacteria [6]. In addition, patients cannot drink and eat, their oral self-cleaning ability is reduced, oral hygiene conditions are reduced, dental plaque is increased, it is difficult to remove, and it becomes a reservoir for VAP pathogens. In addition, patients with mechanical ventilation through orotracheal intubation due to their own resistance weakened, the body's defense function is impaired [7]. Gram-negative bacteria (GNB) are easily colonized in the oropharynx, and the oropharyngeal flora can become pathogenic bacteria when entering the lower respiratory tract [8]. Some scholars have found that the oropharyngeal flora of hospitalized patients often changes after 48 hours. The most prominent is the significant increase in the proportion of GNB colonization. Therefore, for mechanically ventilated patients, reducing oropharyngeal bacterial adhesion, colonization, and aspiration to the lower respiratory tract is effective in preventing VAP [9]. Traditional oral care methods have their inherent limitations, such as the single oral care solution and oral care methods, resulting in poor oral care effects. In order to improve the effect of oral care, our hospital uses a method of combined washing with a modified concentration ratio nursing solution for clinical research [10]. It was found that the improved oral care can effectively improve the cleanliness of oral care and reduce the number of dental plaque in the oral cavity. This is because the improved ratio of oral care solution contains sodium bicarbonate and hydrogen peroxide solution in the corresponding proportions, which can more effectively soften and dissolve the blood crust and sputum adhering to the teeth and gums and then rinse with isotonic saline. The oral cavity can effectively remove the residues in the dead corners, reduce the amount of residual dental plaque in the oral cavity, and improve the cleanliness of the patient's oral cavity [11].

The results of this study showed that after the end of nursing, the oral bacterial flora of the observation group was significantly lower than that of the control group at 8 h, 16 h, and 24 h after intubation. At present, clinical oral care for patients with oral endotracheal intubation often pays attention to postintubation care but does not pay attention to oral cleaning intervention before intubation, ignoring the first pass of bacterial invasion [12]. This study is aimed at improving the shortcomings of ignoring oral cleaning before tracheal intubation in clinical practice. The oral cavity is scrubbed within 30 minutes before intubation to strengthen oral cleaning before intubation. The aim is to reduce the growth and reproduction of pharyngeal bacteria and the oral cavity caused by intubation and thus the risk of bacteria entering the lower respiratory tract [13]. Before nursing, there was no statistically significant difference in the oral bacterial flora of the two groups of patients in this study after oral endotracheal intubation and mechanical ventilation before oral care. It is considered that patients receiving mechanical ventilation are more severely ill and have decreased resistance, impaired body defense function, weakened oral self-cleaning effect, and massive growth and reproduction of bacteria in the oral cavity [14]. In addition, it may also be related to the sterilization timeliness of 0.1% povidone iodine. Therefore, for such patients with tracheal intubation, it may be more reasonable if the interval between oral care can be shortened [15]. In this study, children's soft-bristled toothbrushes were used to scrub and rinse. Compared with conventional oral scrubs, it can effectively remove plaque bacteria and deep oropharyngeal bacteria in the oral cavity. Here are the following advantages: children's toothbrush is small in size and soft in hair. It can not only brush the interdental space, gingival groove, cheeks, and tongue in place and effectively remove dental plaque bacteria but also make oral secretions and tongue coatings easy to fall off and remove food residues. It ensures comfort, conforms to the daily habits of the patient, and makes it easy for the patient to accept [16]. The flushing method uses liquid to continuously flush the oral cavity, which can not only completely remove the dirt in various parts of the oral cavity and the special parts of the deep part of the oral cavity but also can significantly reduce the adsorption capacity of bacteria on the oropharyngeal mucosa and the wall of the intubation tube and with continuous flushing. Attracting and expelling are of positive significance for the prevention of oral and lung infections [17].

The results of this study indicate that after nursing, the number of patients with oral cleanliness in the observation group was significantly higher than that of the control group. It shows that improved oral care can effectively reduce the number of oropharyngeal bacteria in patients undergoing mechanical ventilation through orotracheal intubation, significantly reduce the incidence of ventilator-related pneumonia, and improve oral cleanliness. Analysis of the reasons may be related to the following links: ① oral scrub before intubation can reduce the adhesion of oropharyngeal bacteria to avoid or reduce the entry of bacteria in the oral cavity into the lower respiratory tract due to the intubation action [18]. ② Compared with conventional scrubbing, the experimental group used a soft toothbrush to scrub and rinse the oral cavity after intubation, which can effectively remove dental plaque and dirt in special parts of the oral cavity. ③ The oral care solution uses 0.1% povidone iodine. Povidone iodine has a high-efficiency and broad-spectrum bactericidal effect. It can kill bacterial spores and propagules, fungi, protozoa, and some viruses and can be used for disinfection of skin and mucous membranes without irritation. In addition, its toxicity is extremely low, the bactericidal power is strong, the effect is long-lasting, it is easily soluble in water, and it is not affected by blood, plasma, pus, soap, and pH [19]. Here are the points to note for improved oral care operation and nursing process: Before washing the patient's mouth, carefully check the intubation balloon for air leakage, avoid oral foreign bodies, secretions, and washing fluid entering the respiratory tract, and prevent lung infection and suffocation other complications [20]. During the flushing process, the patient's condition should be carefully observed. When an abnormality occurs, the nursing staff should immediately stop the flushing and accurately find the cause to ensure that the incoming flushing fluid dosage is the same as the outgoing flushing solution [21]. At the same time, during the operation, the nursing staff must be gentle to prevent damage to the patient's oral mucosa and strictly follow the relevant operating procedures to ensure that the intubation does not shift or other problems [22]. According to the changes in the patient's condition, choose appropriate and improved oral care practices, cultivate the sense of responsibility of nurses, and attach importance to improving the professional operating skills of nurses in daily work. Aspiration is a common complication of patients during the treatment of mechanical ventilation through oral endotracheal intubation. If the bacteria in the oropharynx reach the lungs by suction, they reduce the lung defense mechanisms and do not fundamentally solve the pathogenic bacteria and cause infection. Therefore, in the application of improved oral care methods, the role of the soft bristles of the toothbrush should be fully utilized to completely remove the blood and sputum scabs in the patient's oral cavity [23–27].

This study is aimed at improving the inefficiency and limitations of oral care for patients with clinical oral endotracheal intubation and strengthened early oral cleaning before intubation and oral care after intubation. The results showed that oral cleanliness score, mechanical ventilation time, ICU stay time, and GCS score in the observation group were better than those in the control group. This clinical study concludes the following: compared with conventional oral care methods, early intensive oral care reduces the incidence of VAP in patients with tracheal intubation, alleviates the suffering of patients, and does not increase medical costs. In terms of feasibility, improved oral care is not only simple to operate but can be mastered after short training. In clinical practice, nurses are easy to accept and have operability [28–32]. In terms of methodology, this study excluded patients with heartbeat, respiratory arrest, or other patients who need emergency endotracheal intubation. At the same time, the oral scrub control before intubation was completed within 2 minutes without delaying the timing of the patient's intubation and the rescue effect because physiological studies have proved that the body's own oxygen reserves can maintain the body's 2 min oxygen supply [33–35]. For patients who underwent oral scrub before tracheal intubation, the mask should be pressurized and oxygenated to make SPO2 ≥ 95%, and if necessary, nasal cannula should be given oxygen inhalation during scrubbing.

Since this experiment is still in the preliminary research stage, the sample size is not large enough to compare the methods of oral care and oral care solutions. Therefore, based on the initial results, we should further increase the sample size and expand the grouping of in-depth research in the future to explore a more effective and convenient oral care method for the oral care of patients with oral endotracheal intubation and improve the quality of oral care. Reduce the incidence of VAP as much as possible, so that the improved oral care methods can be better promoted and applied in clinics. In summary, improved oral care can effectively reduce the number of oropharyngeal bacteria in patients undergoing mechanical ventilation through orotracheal intubation and significantly reduce the incidence of ventilator-associated pneumonia, improve oral cleanliness, and reduce mechanical ventilation time, which is more helpful and improves the quality and effectiveness of oral care.

## 5. Conclusion

Oral care can effectively reduce the number of bacteria in the oropharynx of patients with mechanical ventilation through orotracheal intubation, significantly reduce the incidence of ventilator-associated pneumonia, and improve the quality and effectiveness of oral care.

## Figures and Tables

**Figure 1:** The research procedure.

**Table 1:** Comparison of oral bacterial flora between the two groups ($\bar{x}\pm s$).

Group	After intubation 8 h		After intubation 16 h		After intubation 24 h	
	Care before	Care after	Care before	Care after	Care before	Care after
Control group (50)	5.60 ± 1.18	5.57 ± 0.29	5.84 ± 1.21	5.65 ± 0.35	5.91 ± 1.48	5.33 ± 0.21
Observation group (50)	5.65 ± 1.27	5.27 ± 0.35	5.83 ± 1.28	5.17 ± 1.23	5.87 ± 1.49	5.15 ± 0.19
*F*	-0.204	4.667	0.040	2.654	0.135	4.494
*P*	0.839	<0.001	0.968	0.009	0.893	0.001

**Table 2:** Oral cleanliness and incidence of ventilator-associated pneumonia in the two groups ($\bar{x\pm s}$).

Group	Oral cleanliness			The incidence of ventilator-associated pneumonia		
	I°	II°	III°	Early onset	Late onset	Total incidence
Control group (50)	15 (30.00)	13 (26.00)	22 (44.00)	3 (6.00)	9 (18.00)	12 (14.00)
Observation group (50)	5 (10.00)	14 (28.00)	31 (62.00)	2 (4.00)	3 (6.00)	4 (8.00)
*χ* ^2^	8.294			/	/	4.762
*P*	0.016			/	/	0.029

**Table 3:** Mechanical ventilation time, ICU hospitalization time, and mortality rate of the two groups of patients ($\bar{x\pm s}$).

Group	Oral cleanliness score	Mechanical ventilation time (d)	ICU hospital stay (d)	Mortality rate (%)	GCS score
Control group (50)	19.25 ± 3.82	18.31 ± 4.51	24.31 ± 4.51	16	9.34 ± 1.25
Observation group (50)	15.27 ± 4.31	14.30 ± 3.52	19.30 ± 6.52	12	13.33 ± 2.24
*χ* ^2^ */t*	4.887	4.956	4.469	0.794	-10.999
*P*	<0.001	<0.001	<0.001	0.373	0.001

## Data Availability

No data were used to support this study.
